The article "CircKMT2E Participates in Osteoarthritis through Promotes Apoptosis of Chondrocytes Via Sponging miR-140-5p to Activate TLR4" was retracted in 2023. Reasons: signs of a paper mill; suspected computer-generated content; unreliable results or conclusions; concerns about the data.

# CircKMT2E Participates in Osteoarthritis through Promotes Apoptosis of Chondrocytes Via Sponging miR-140-5p to Activate TLR4

**DOI:** 10.1155/2022/2957844

**Published:** 2022-09-15

**Authors:** Yong He, Fubo Zhou, Xianqiang Cheng

**Affiliations:** ^1^Department of Orthopedics, Hubei Hospital of Traditional Chinese Medicine, Wuhan, Hubei 430074, China; ^2^Department of Trauma Orthopedics, Laiyang Central Hospital, Yantai, Shandong 265200, China

## Abstract

**Objective:**

To explore the latent pathogenesis of circRNAs in osteoarthritis (OA), as well as their function mechanism.

**Methods:**

The murine chondrocytes with and without OA were involved and used for in-depth sequencing. Herein, we carried out subsequent bioinformatics analysis to disclose the expression pattern, characteristics of circRNAs based on gene ontology, and the KEGG pathway analyses. Then sequencing data were used to deduce the interaction between circRNA and miRNA. The potential miRNA response elements for the annotated circRNAs and relevant target genes were forecasted on the basis of TargetScan and miRanda. For chondrocytes, the effect of the overexpression of the screened circRNA for apoptosis was spotted by flow cytometry as well as Western Blot.

**Results:**

466 diverse circRNAs in the 23,787 spotted circRNAs were both significantly and differentially transcribed. CircKMT2E was upregulated more than two folds in chondrocytes with OA compared with normal tissues, exhibiting an expression trend opposite to miR-140-5p. We disclosed that circKMT2E could possess mutual effect with miR-140-5p by way of AGO proteins. Thus, circKMT2E was verified to have functioned as a molecular sponge targeting miR-140-5p. Therefore, circKMT2E may be at work in the pathogenesis of OA. Further, the sponge connection between circKMT2E and miR-140-5p was proved on the basis of a dual-luciferase reporter assay. Besides, miR-140-5p was speculated can bind TLR4 by bioinformatics analysis. Further PCR analysis found the relative expression level of TLR4, caspase-3, and Bax in the OA groups presented significant upregulation. Overexpression of circKMT2E can promote apoptosis of chondrocytes.

**Conclusion:**

The upregulation of circKMT2E is involved in the chondrocyte apoptosis of the pathogenesis of OA through activation of TLR4 by the sponge function of miR-140-5p.

## 1. Introduction

Osteoarthritis (OA) as a sort of degenerative disease that occurs in joint that causes decreased quality of life or even physical disability, is mainly depicted by the gradual inflammatory undermine of articular cartilage [1, 2]. The overall sum of patients subjected to OA has been reckoned to exceed at least 250 million globally. Besides, the number of sufferers is still augmenting promptly and continuously [3]. OA affects approximately 80% of the population that aged more than 60 years, which also occupies a great proportions for numerous hospitalizations annually in the many under-development and developed world [1]. However, the clinical therapeutic effect of OA is still not ideal. As a consequence, to disclose novel theoretical contribution targets to the prevention as well as the treatment of OA, it is indispensable to intensify the studies that focus on this relevant domain.

Since chondrocytes are the single cells that exist in articular cartilage, chondrocytes play a role in the progression of pathology of OA, especially by relying on both cytokine production and apoptosis. [4, 5] Chondrocytes widely express toll-like receptors (TLRs), which are a subgroup of receptors possessing the capacity for pattern-recognition and can discern intruding microorganisms as well as harmful endogenous substances in order to induce immune reactions. In the midst of TLRs, TLR4 is crucial for apoptosis and the inflammatory response of chondrocytes. [2].

miR-140 as a kind of chondrocyte-specific miRNAs, is indispensable for the proliferation of endochondral bone. If miR-140 becomes deficient, osteal deformity as well as dwarfism would be given rise to [6]. The miR-140 gene encodes three subtypes of microRNAs, miR-140-3p.2, miR-140-3p.1, and miR-140-5p [6]. However, the crucial mRNAs that miR-140 miRNAs physiologically target remain undefined. Yang [7] recently reported that apoptosis and cellular inflammation in lipopolysaccharide-induced WI-38 cells can be inhibited via miR-140-5p/TLR4 pathway when long noncoding RNA H19 is silenced. However, the interaction between miR-140-5p and the TLR4 pathway in OA has not been explored yet. In order to reveal the latent pathogenetic process of OA as well as to ascertain the function of miR-104 in chondrocytes, in-depth sequencing was used for the murine cartilage tissue with and without OA.

## 2. Methods

### 2.1. In-Depth Sequencing Data

The in-depth transcriptomic data of both healthy and OA murine cartilaginous tissues were downloaded from the NCBI bioproject database with accession numbers PRJNA798112 and PRJNA817158, in which, after stratified sampling, three healthy samples and three OA samples were enrolled in this research. Wild male C57BL/6 mice were used for the experimental procedures when aged 8 weeks old. The destabilisation of the medial meniscus incised the right knee of the mice with a patella tendon in the middle, and the tendon between the medial meniscus and the tibial plateau was cut in virtue of a diminutive surgical scissors. For the control group, only arthrotomy was implemented, namely medial meniscotibial ligament cutting was exempted.

### 2.2. Differential Gene Expression Analysis

Sequence reads with high quality were then matched to the reference transcriptome using the STAR software (v2.5.1b) [8]. CircRNAs were discerned with DCC software and annotated on the basis of the circBase database as well as circ2Traits. CircRNAs that were differentially expressed between above-mentioned two groups were recognized on the basis of *t*-test. The *p* value was corrected using the Benjamini & Hochberg method. [9] The differential circRNAs were scanned and outputted so long as fold-change ≥2.0 as well as *p* value ≤0.05.

### 2.3. GO and KEGG Analyses

The enrichment analyses on the basis of GO as well as KEGG that aims to disclose differentially expressed circRNAs were implemented. GO is a methodic and organized database in order to depict both genes and their products. It not only covered molecular function but also revealed biological process as well as cell component. With the help of the pathway analysis from KEGG, the signaling pathways that containing circRNAs as well as their biological functions can be inferred. The relevant *p* value was computed on the basis of Fisher's exact test (threshold value being 0.05).

### 2.4. OA-Related Candidate circRNA Analysis

The abundance of circRNAs was calculated by Ballgown and computed by FPKM. The threshold value of FPKM in each group was 0.5, which means the circRNA would be deemed as expressed in this group if FPKM >0.5. For circRNAs expression, Student's *t*-test was applied on the basis of GraphPad Prism 8.0 to compute the significance for differences.

### 2.5. Interaction Network Analysis of circRNA-miRNA and Target Gene

The underlying miRNA reaction elements for the annotated circRNAs and target gene were predicted using the custom-written software which on the basis of both TargetScan and miRanda (Cloud-seq Biotech, Shanghai, China). CircPrimer1.2 (https://www.bioinf.com.cn/) and the UCSC genome browser were used to annotate the structure of circKMT2E and its positions on parental genes, respectively. The CircMir1.0 software, on the basis of the miRanda 2010 deliver (https://www.microrna.org/microrna/getDownloads.do) and RNAhybrid-2.1.2, was applied to annotate putative bundling situations of miR-140-5p on circKMT2E transcripts.

### 2.6. Cell Culture and Transfection

The human primary chondrocytes cells (HUM-iCell-s018, iCell, China) were cultured in Primary Chondrocyte Culture System (PriMed-iCell-020, iCell, China). CircKMT2E mimics and circRNA control were synthesized by Aksomics Inc. (Shanghai, China). The aforementioned circRNAs (20 nM) were transfected into the human primary chondrocytes cells (2 × 10^6^) on the basis of Lipofectamine 2000 (11668030, Thermo Fisher, USA) at 37°C. Afterwards, the transfected cells, after 48 h transfection, were reaped to accomplish the following procedures.

### 2.7. Dual-Luciferase Reporter Assay

To validate the direct combination between miR-140-5p and circKMT2E, the dual-luciferase reporter assay was applied. Multiple cloning sections of the psiCHECK-2 plasmid were subcloned according to the saltatory sequences as well as the wild-type of circKMT2E. Accordingly, the target-section that involves the aforementioned luciferase reporter carrier, in company with miR-140-5p mimics or blank controls of miRNA, was transfected simultaneously into human primary chondrocyte cells in virtue of Lipofectamine 2000 (11668030, Thermo Fisher, USA). After 48 hours, we spotted the fluorescence activities on the basis of the Luc-Screen Assay System (T1033, Thermo Fisher, USA), and computed the comparative fluorescence activities.

### 2.8. qRT-PCR

Total RNAs were extracted on the basis of TRIzol (15596018, Life Technologies, USA). Whereafter, the density of extracted RNAs was assessed based on NanoDrop (ND-ONE-W, Thermo Fisher Scientific, USA), as well as the value of OD260/OD280 within 1.8–2.1. Then, cDNAs were compounded on the basis of the SuperScript Kit (18080093, Invitrogen, USA). Further qRT-PCR was carried out on the ViiA 7 Real-time PCR System (4453536, Applied Biosystems, USA) on the basis of the PowerTrack SYBR Green Master Mix (A46012, Applied Biosystems, USA). Relevant primers were engineered by primer 5.0 on the basis of the longitudinal transcripts [10]. The relative content of circRNAs as well as miRNAs was computed on the basis of the 2^−ΔΔCT^ method. Beta-actin was used as an internal reference. Based on the GraphPad Prism 8.0, we used Student's *t*-test to ensure the significant differences for circRNAs.

qRT-PCR was applied to check the expression extent of apoptosis-related gene, circRNAs with differential expression, as well as miR-23b-3p. Involved primer sequences: beta-actin: 5′-GAACCGACTTCTCCCCTTGT-3′ and 5′-TCGTCTGTTAGGTGGATGCTT-3′. circKMT2E: 5′-TGACCTCCTTCGCCACTTAC-3′ and 5′-CATAACAGCGTCACCACAGC-3′. miR-140-5p: 5′-AAGAGACTGGGGTGTGGAAA-3′ and 5′-TCTGAAGTTTTCCATTTCTCTGC-3′. TLR4: 5′-GGGATCACATTGCCAGGGAT-3′ and 5′-CAGTGCGTGTCGTGGAGT-3′. Caspase-3: 5′-CTCGCTTCGGCAGCACA-3′ and 5′-AACGCTTCACGAATTTGCGT-3′. Bax: 5′-CAAAGGGAATACATTGCCAGA-3′ and 5′-TGTGGCCAACTGCTGAAA-3′.

### 2.9. Western Blot

Total protein, with the help of RIPA buffer including protease inhibitor, was extracted. To explore the protein concentrations, the BCA protein assay kit (Thermo Fisher Scientific, USA) was applied in this study. Proteins (∼50 *μ*g) went through electrophoresis on the basis of 10% SDS-PAGE, therewith, transferred proteins onto PVDF membranes. Then membranes were blocked at room temperature for 2 h on the basis of 5% bovine serum albumin (Abcam, USA). Then, all samples were soaked by primary antibodies all night at 4°C and then soaked by HRP-conjugated secondary antibodies at 26°C for 2 h. Eventually, the enzyme-linked chemiluminescence kit (Millipore, Billerica, MA) and CD-touch (Bio-Rad, Hercules, CA, USA) were applied to photograph the blots which can be quantified on the basis of Image Lab software. Above-mentioned antibodies were purchased from Abcam.

## 3. Results

### 3.1. The Landscape of circRNAs in OA and Healthy Tissues

To grasp the managing mechanisms of circRNAs in OA, the expression pattern of circRNAs in chondrocytes was disclosed in this study. In short, we downloaded RNA data of total RNAs from NCBI, which included the control group and OA group (3 replicates, respectively). Then, we used a computational program on the basis of the Ensembl transcriptome GTF file as well as the DCC software to ascertain circRNAs.

Based on unique junction reads ≥123,787, diverse circRNAs were detected across all samples (Figures 1(a) and 1(b)). For the OA group, 17,345 diverse circRNAs were disclosed. In addition, 14,491 circRNAs were revealed in the control group. By searching overt data in circBase, we found 15,050 (63.3%) of all circRNAs were in accordance with the database. On the other hand, 8,737 (36.8%) circRNAs were first disclosed (Figure 1(a)). After functionally annotating circRNAs in the genome, 76.7% of detected circRNAs were situated in protein-coding exons. Besides, the remaining circRNAs were respectively sided with introns, antisense, and intergenic, as well as sense overlapping regions (Figure 1(c)). In addition, the length distributional characteristic of exon-related circRNAs was presented with 560 nt as the median length (Figure 1(d)).

### 3.2. CircRNAs with Differential Expression in the OA Group

The circRNAs with differential expression in the OA group were subsequently analyzed. In this research, discriminating criteria were respectively set as fold-change ≥2 and *p* < 0.05 for the purpose to seek circRNAs that differentially expressed (Figures2(a) and 2(b)). In contrast to the control samples, 466 circRNAs that differentially expressed were found within the OA tissues. Therein, 200 appeared upregulated while 266 appeared downregulated. Additionally, the connection of differential fold alterations between the OA and control group was analyzed, which found an advanced correlation in circRNAs with significant down-regulation rather than circRNAs with significant upregulation (Figure 2(b)). However, circKMT2E presented remarkable upregulation. Consequently, we further inspected circKMT2E, a downregulated circRNA, to probe into its' managing capacity in OA formation.

### 3.3. CircKMT2E Was Highly Expressed in Chondrocytes with OA and can Bind to miR-140-5p

High-throughput sequencing data disclosed that circKMT2E was also markedly piled up in the chondrocytes with the OA (Figures 3(a) and 2(a)). As a consequence, we chose circKMT2E, a potential biomarker, to establish forward research. According to the StarBase database which is based on CLIP-Seq laboratorial approaches, we took notice that circKMT2E could unite to miR-140-5p with the help of AGO proteins. The mutual relation between circKMT2E and miR-140-5p was recognized on the basis of a dual-luciferase reporter assay, which can verify the binding capacity between circRNAs and miRNAs. In contrast to the control group, the luciferase content (Figure 4) was markedly descended by miR-140-5p in the circKMT2E -WT group. On the other hand, the luciferase activity was nearly unvaried in the circKMT2E-MUT group in contrast to the control group. Besides, circKMT2E significantly increased in chondrocytes with the OA in contrast to the controls, while miR-140-3p markedly decreased in chondrocytes with OA in contrast to the controls (Figures 2(a) and 2(d)). As a consequence, miR-140-5p leaned to present negative relationship to circKMT2E (Figure 2(b)). Since circKMT2E was disclosed to directly combine with miR-140-5p, we deduced that circKMT2E may sponge miR-140-5p as a ceRNA and take part in the advancement of OA.

### 3.4. Functional Deduction of the Target Genes of circRNAs with Significant upregulation

CircRNAs could play the part of the sponges of miRNA, through which they can manage the expression of interrelated host genes. [10] To deduce the underlying capacity of filtered downregulated circRNAs in the OA, Kyoto Encyclopedia of Genes and Genomes (KEGG) as well as gene ontology (GO) enrichment analyses were performed (Figure 5). Metabolism was analyzed to be one of the most significant functions in the biological process. The functions of host gene which participated in a series of cellular physiological functions, for example, the governance of growth, apoptosis, and stress response. GTPase activator activity, bridging and protein binding in the molecular functions of the analysis of GO enrichment disclosed that circRNAs with significant as well as differential expression, to some extent, could manage cellular apoptosis or proliferation by taking part in cellular signaling pathways. The analysis on the basis of KEGG pathway revealed that their parental genes of circRNA that possess differential expression were related to the longevity regulating pathway, AMPK pathway, as well as mTOR signaling pathway, which acted as a key role in apoptosis process as well as cellular oxidative stress [9, 10]. These results discovered cues that upregulated circRNAs could take part in the development as well as formation of the OA based on various channels.

### 3.5. CircKMT2E Is Associated with the Apoptosis of Chondrocytes in the Pathogenesis of OA via miR-204-5p Sponge Function

To probe into the potential connection between the identified circRNAs and miRNAs during the development of OA, we took circKMT2E (chr3: 150903117-150911453+) as an example and predicted target mRNAs of the five leading miRNAs binding to circKMT2E using TargetScan and miRanda [9, 10]. We annotated the relation in a circRNA-miRNA-mRNA network that was mapped by the cytoscape software (Figure 6). As the figure shows, miR-140-5p was discovered to target TLR4, ALDH3A2, and SOD2. Among these target genes, TLR4 has an intimate relationship with apoptosis. As a result, we detected the relative expression levels of TLR4, caspase-3, and Bax in the normal and OA groups by PCR (Figure 7). Caspase-3 and Bax were both upregulated in the OA group, which suggested circKMT2E is associated with the apoptosis of chondrocytes in the pathogenesis of OA via miR-204-5p sponge function.

### 3.6. Overexpression of circKMT2E can Promote Apoptosis of Chondrocytes

To verify the promoting function for apoptosis of circKMT2E *in vitro*, we used human primary chondrocytes cell, respectively, transfected by circKMT2E and circRNA-control to detect apoptosis rate using flow cytometry and apoptosis-related protein using Western blot. As flow cytometry results disclosed that the upregulation of circKMT2E significantly enhanced the apoptosis rate of chondrocytes cells, while no significant differences were found between the circRNA-control group and the blank control group (Figure 8). In addition, the results of Western Blot disclosed that the overexpression of circKMT2E significantly increased cyT-C and Bax and significantly decreased the expression level of Bcl-2. Besides, the expression of Bcl-2, Bax, and Cyt-C were found to have no significant difference in the circRNA-control group compared with the blank control group.

## 4. Discussion

Synovium, as one of the most crucial components of the joint system, is formed by loose connective tissue. The core functions of the synovium include weakening joint surface friction, secreting synovial fluid, offering nutrients to articular cartilage, restraining joint adhesion, restraining cell fragments in the joint cavity, and assimilating miscellaneous metabolites. When stress of injuries, such as trauma, degeneration, infection, and rheumatism, comes to the joint, the partly undesirable inflammatory reaction of the synovium will be stimulated to take part in the purpose of repairing the injury to the articular cartilage. It is found that OA synovitis usually presents chronic as well as low-grade inflammation as the dominating feature, which may intimately come to the pathogenetic process of the cartilage damage of OA. Accordingly, endeavoring to adjust the condition and circumstances of synovitis in order to rebuild the local microenvironment of the OA joint as well as accelerate the repair progress of chondrocytes is promising to serve as a viable approach for the clinical treatment of OA. Whereas, the formation progress and molecular mechanism of OA synovitis remains unclear.

Previously, plenty of researches have disclosed that, during the process of OA, synovial tissue was motivated to generate inflammatory responses and ultimately to generate and contribute to the constitution of chronic synovitis by the cellular fragments from lifeless chondrocytes and degradative cartilage matrix. [11]. Therefore, apoptosis of chondrocytes may be a key process in the constitution of chronic synovitis of OA on the basis of motivating synovial inflammatory cells. Recently, Bao et al. [12] found that rapamycin can preserve chondrocytes from IL-18-induced apoptosis as well as improve OA in rats. Wang et al. [13] revealed that aucubin can preserve chondrocytes from IL-1*β*-induced apoptosis as well as inhibit OA. Ding et al. disclosed that miR-93 can inhibit cellular apoptosis of chondrocytes as well as inflammation occurs in OA on the basis of targeting the TLR4/NF-*κ*B signaling pathway.

In this study, we first disclosed the expression patterns of circRNAs in murine chondrocytes related to OA. In murine chondrocytes with OA, circKMT2E was disclosed to be the most significant upregulated circRNA. Further study revealed circKMT2E possesses a negative correlation with miR-140-5p, which is one of the chondrocyte-specific miRNAs and is indispensable for normal endochondral bone proliferation in mice. PCR also verified the enlarged expression of circKMT2E and diminished expression of miR-140-5p in OA tissue.

Inflammation-induced catabolism includes cell dedifferentiation, matrix metalloproteinase reaction, restraint the expression of type II collagen as well as aggrecan core protein are firmly dominated by TLR-dependent immune reaction. [14, 15] For humans, a series of 10 different type I transmembrane receptors that possess specificity for diverse kinds of PAMPs constitute the TLR family [16, 17]. A few TLRs could also perceive host-derived molecules which are fruited when injuries occurr to tissues, alleged damage-associated molecular patterns. Among these TLRs, TLR4 senses more damage-associated molecular patterns than others. [14] TLR4 is highly expressed in chondrocytes, synoviocytes, and osteoblasts, supporting an important role in the physiology as well as pathology of joint tissues [16, 18]. For example, TLR4 can modulate apoptosis through the NF-*κ*B pathway. [19, 20].

Therefore, the relative expression levels of TLR4, caspase-3, and Bax in the normal and OA groups were detected by PCR. TLR4 and these two apoptosis-related proteins all presented significant upregulation in the OA group. To moreover check on the circKMT2E/miR-140-5p/TLR4 regulatory pathway, our research team performed a dual-luciferase reporter assessment to confirm the combinative connection between circKMT2E and miR-140-5p, they used transfected cells to verify the ability of circKMT2E to promote apoptosis. Wang et al. [21] previously found that knockdown of LINC01385 can inhibit the progression of OA on the basis of adjusting the microRNA-140-3p/TLR4 axis. Thus, it can be deduced that upregulated circKMT2E in chondrocytes with OA may be involved in the apoptosis of chondrocytes by targeting TLR4 via the sponge function to miR-140-5p. Although the exact mechanisms need further validation, our study found that the circRNAs that showed differential expression take part in the pathogenesis of OA, which can provide a novel target for the therapy of OA.

This study has a few limitations. First, the visualized results of the overexpression study were not carried out owing to our limited laboratory conditions. Second, the specific signaling pathway of chondrocyte apoptosis were not further explored. Third, the murine gene knock-out research were not involved.

## 5. Conclusion

In this present study, differentially expressed circRNAs in murine chondrocytes with OA were analyzed. We preliminarily disclosed the sponge interaction between miR-140-5p and OA related circKMT2E. The upregulation of circKMT2E may be involved in the chondrocyte apoptosis of OA through activating TLR4 by sponging miR-140-5p.

## Figures and Tables

**Figure 1:** Spotted circRNAs in the OA group and healthy tissues. (a) The consistency among the control group, OA, as well as CircBase for circRNAs. (b) The amount of circRNAs as well as junction reads discerned in OA as well as the control group. (c) The positional feature of spotted circRNAs. (d) The distributional characteristic of length for exon-related circRNAs.

**Figure 2:** CircKMT2E was highly expressed in chondrocytes with OA and can bind to miR-140-5p. (a) PCR results of circKMT2E in the chondrocytes with OA. (^*∗∗∗*^, *p* < 0.001). (b) On the basis of the relative expression, the connection between circKMT2E and miR-140-5p probed by FPKM analysis disclosed a negative correlation. (*p* < 0.05). (c) CircKMT2E was situated between the second and fourth exons in its host gene. (d) Confirmation of miR-140-3p in the control and OA groups by PCR.

**Figure 3:** Differentially expressed circRNAs in the OA as well as the control group. (a) The volcano plot of the OA group for spotted circRNAs. (b) The Venn diagram presents circRNAs with differential expression in the OA as well as the control group. (c) The positional feature of circRNAs in chromosome. The most outer tier discloses the chromosomal situation of the circRNAs. By contrast, from the outside to the most inside of the inner circles, they disclose the distribution characteristic of all circRNAs in the OA as well as the control group, circRNAs with differential expression in the OA group, and circRNAs that possess differential expression in the control group.

**Figure 4:** Dual-luciferase reporter assay for circKMT2E as well as miR-140-5p.

**Figure 5:** Enrichment analysis on the basis of GO (a) as well as KEGG (b) for parental genes of differentially expressed circRNAs. The enriched terms of GO as well as KEGG connected with the OA pathological process were ordered on basis of the enrichment score, namely-log10 (*p* value).

**Figure 6:** A derived circRNA-miRNA-mRNA interaction map based on StarBase and TargetScan. The violet arrowheads stand for circRNAs, the green circles stand for OA-associated miRNAs, and the blue units stand for the target genes with the most significant correlation.

**Figure 7:** The relative expression levels of TLR4, caspase-3, and Bax in the normal and OA groups by PCR.

**Figure 8:** In human primary chondrocytes cells, the overexpression targets of miR-140-5p could promote apoptosis. (a-b) the results of flow cytometry disclosed that the overexpression of miR-140-5p can significantly increase the apoptosis rate (c-d). The Western Blot results of human primary chondrocytes cells presented that the overexpression of miR-140-5p could outstandingly augment the expression levels of Cyt-C and Bax and outstandingly reduce the expression level of Bcl-2.

## Data Availability

The labeled dataset used to support the findings of this study is available from the corresponding author upon request.
